RETRACTED

# A Review of Bile Acid Metabolism and Signaling in Cognitive Dysfunction-Related Diseases

**DOI:** 10.1155/2022/4289383

**Published:** 2022-03-11

**Authors:** Ze-Bin Weng, Yuan-Rong Chen, Jin-Tao Lv, Min-Xin Wang, Zheng-Yuan Chen, Wen Zhou, Xin-Chun Shen, Li-Bin Zhan, Fang Wang

**Affiliations:** ^1^School of Traditional Chinese Medicine & School of Integrated Chinese and Western Medicine, Nanjing University of Chinese Medicine, Nanjing, China; ^2^College of Food Science and Engineering/Collaborative Innovation Center for Modern Grain Circulation and Safety/Key Laboratory of Grains and Oils Quality Control and Processing, Nanjing University of Finance and Economics, Nanjing, China; ^3^The Innovation Engineering Technology Center of Chinese Medicine, Liaoning University of Traditional Chinese Medicine, Shenyang, China

## Abstract

Bile acids are commonly known as one of the vital metabolites derived from cholesterol. The role of bile acids in glycolipid metabolism and their mechanisms in liver and cholestatic diseases have been well studied. In addition, bile acids also serve as ligands of signal molecules such as FXR, TGR5, and S1PR2 to regulate some physiological processes in vivo. Recent studies have found that bile acids signaling may also play a critical role in the central nervous system. Evidence showed that some bile acids have exhibited neuroprotective effects in experimental animal models and clinical trials of many cognitive dysfunction-related diseases. Besides, alterations in bile acid metabolisms well as the expression of different bile acid receptors have been discovered as possible biomarkers for prognosis tools in multiple cognitive dysfunction-related diseases. This review summarizes biosynthesis and regulation of bile acids, receptor classification and characteristics, receptor agonists and signaling transduction, and recent findings in cognitive dysfunction-related diseases.

## 1. Introduction

Bile acid (BA) is an important component of bile, which is stored in the gallbladder and released into the intestinal lumen for lipid digestion in response to food intake. The enterohepatic circulation of BAs is carried out 6 to 15 times per day, and about 95% of BAs in the intestinal lumen are passively or actively reabsorbed and then returned to the liver through the portal vein circulation with 0.4 to 0.6 g of BAs excreted from the stool. What is more, BAs are also acted as steroid hormones to regulate metabolic processes by interacting with BA receptors such as farnesoid X receptor (FXR), cell membrane surface receptor-G protein-coupled receptor (TGR5), and sphingosine-1-phosphate receptor 2 (S1PR2) to initiate downstream signaling pathways [1–3]. In recent years, BAs have been found as metabolic regulators and nutrient sensors in regulating glucose and lipid metabolism, appetite, and immune response [4–6]. Surprisingly, emerging evidence showed that BAs might be a novel regulator in the physiological and pathological processes of the nervous system. Different kinds of BAs and their receptors have been found in the brains of humans and rodents. Specific BA like ursodeoxycholic acid (UDCA) and tauroursodeoxycholic acid (TUDCA) has been proved to exhibit novel neuroprotective properties and has been utilized in a clinical trial [7–9]. In addition, with the comprehensive research on the “gut-brain” axis in recent years, more and more studies have found that BAs, as a metabolite closely related to the intestinal flora, may act as a “messenger” in the “gut-brain” axis [10, 11]. Alteration in BA metabolism and its associated receptors have also been found in the patients or animal models of cognitive dysfunction-associated diseases in the latest research [12, 13]. Therefore, in this review, we focus on the current studies and latest findings on BA anabolism, the signaling and related mechanism of BA and its receptors in cognitive dysfunction-associated diseases, and the intervention of related drugs in cognitive dysfunction by regulating BA metabolism.

RETRACTED

## 2. Synthesis and Metabolism of BA

### 2.1. Biosynthesis of BAs

The homeostasis of cholesterol in vivo is mainly maintained by the synthesis and efflux of cholesterol, in which BA synthesis through a series of enzymatic reactions is the main pathway of cholesterol metabolism. About 500 mg of cholesterol is converted into BAs in the hepatocytes surrounding the central hepatic vein (perivenous hepatocytes) of an adult every day [14]. There is a classical and alternative pathway for BA synthesis [15]: the classical pathway is the primary path for BA synthesis which produces about 75% of the total BA. It is catalyzed by a family of unique cytochrome P450 enzymes of a 14-step enzymatic reaction located in the cytoplasmic microsomes, mitochondria, and peroxisomes. The reaction was initiated via the rate-limiting enzyme 7*α*-hydroxylase (CYP7A1) [16], which catalyzed cholesterol into 7*α*-hydroxycholesterol. Then, it was catalyzed by 3*β*-hydroxy-*δ*5-C27 steroid dehydrogenase (3*β*-HSD) in the microsomes to generate *α*-hydroxy-4-cholesten-3-one (7*α*-hydroxy-4-cholesten-3-one, C4) and then catalyzed by sterol 12*α*-hydroxylase (CYP8B1), resulting in metabolic products of cholic acid (CA). The alternative pathway only accounts for about 9% of total bile acid synthesis in human hepatocytes. When the classical pathway is suppressed, the alternative pathway is upregulated and becomes the main bile acid synthesis pathway in some pathological conditions like patients with liver disease. It is initiated by mitochondrial sterol 27-hydroxylase (CYP27A1) which is distributed in multiple tissues and macrophages [17, 18]. Cholesterol was oxidized via CYP27A1, converting into 27-hydroxyl cholesterol and then to 3*β*-hydroxy-5-cholinic acid. 3*β*-Hydroxy-5-cholinic acid is catalyzed by a nonspecific oxysterol 7*α*-hydroxylase (CYP7B1) [19] for the formation of 3*β*, 7*α* -dihydroxy-5-cholinergic acid, followed by HSD3B1/3B2 to synthesize 7a-hydroxy-3-oxo-4-cholesterol acid. These metabolites are finally transported to the liver for the formation of CA and CDCA [20–22]. For rodents like mice [23, 24], CDCA is converted to *α*-muricholic acid (*α*-MCA) by the enzyme sterol-6b-hydroxylase (CYP2C70), and *α*-MCA can be epimerized (isomerized) to a 7*β*-OH group to form *β*-MCA. Besides, CDCA can also be epimerized to form UDCA (more details are shown in Figure 1).

RETRACTED

### 2.2. Gut Microbiota in BA Metabolism

The gut microbiota plays a key role in BA synthesis, modification, and signal transduction. Most of the BAs (about 95%) secreted into the intestine by the gallbladder are actively reabsorbed in the ileum and participate in the enterohepatic circulation of BAs. Another 5% of unabsorbed primary BAs in the intestinal tract are converted to secondary BAs by the gut microbiota through deconjugation, dehydroxyl dehydrogenation, and isomerization [25, 26]. It has been demonstrated that the gut microbiota affects BA diversity in a farnesoid X receptor- (FXR-) dependent manner. The FXR affects primary BA synthesis by inhibiting the activity of CYP7A1 via inducing and binding to the fibroblast growth factor 15/19 (FGF 15/19) in ileum epithelial cells [27, 28]. The metabolism of BA in the intestinal tract requires the participation of intestinal microbial enzymes, of which bile salt hydrolases (BSH) are the main enzyme. BSH can convert conjugated BAs into unconjugated BAs to provide protection and colonization for some gut bacteria. The BSH can directly change the BA structure through sulfonation, oxidation, isomerization, dihydroxylation, and other catalytic modifications. Changes in gut microflora also alter the expression level of BSH, thus affecting the composition of the host BA pool and BA signaling [10, 25] (more details are shown in Figure 1). In the human intestinal tract, deoxycholic acid (DCA) is mainly generated by CA, and lithocholic acid (LCA) and UDCA are generated by CDCA. The major secondary BAs in mice are murine deoxycholic acid (MDCA) and porcine deoxycholic acid (HDCA) which are generated by *α*-MCA and *β*-MCA. Intestinal flora involved in BA metabolism and their modes of action is shown in Table 1.

RETRACTED

### 2.3. Enterohepatic Circulation of BAs

After being synthesized in the liver, BAs are pumped into bile into the small intestine by bile salt export pump (BSEP) and multidrug resistance-associated protein 2 (MRP2). After eating, the gallbladder contracts and secretes BAs into the intestine. A small portion of BAs can be absorbed by the duodenum through passive absorption. About 95% of BAs are actively ingested in the ileum through the apical sodium-dependent BA transporter (ASBT) at the tip of the brush edge of the small intestine and then enter the small intestinal epithelial cells [40, 41]. After binding with the ileal BA binding protein (IBABP), BAs are secreted into the portal vein by the organic solute transporters alpha and beta (OST*α*/OST*β*). Then, the BAs are reabsorbed by liver cells via Na+-dependent taurocholic cotransporting polypeptide (NTCP) and organic anion transporting polypeptides (OATPs) [42, 43]. The enterohepatic circulation effectively recovers about 95% of BAs and minimizes fecal and urinary BA excretions which is an effective way of reabsorption and circulation that causes the total bile salt pool to undergo 4-12 cycles per day. [44] (more details are shown in Figure 2).

### 2.4. Negative Feedback Regulation Mechanism of BA Synthesis

The biosynthesis of BAs is regulated by a negative feedback mechanism (more details are shown in Figure 2). There are two known pathways: the intestinal FXR/FGF19/FGFR4 pathway [14] and the hepatic FXR/SHP pathway [45, 46]. In the liver, excess BAs activate FXR, which induces the expression of the target gene SHP. SHP inhibits the gene expression of CYP7A1 and reduces BA production by binding with liver receptor homologue-1 (LRH-1). SHP can also bind to hepatocyte nuclear factor 4*α* (HNF4*α*), which can inhibit the interaction between HNF4*α* and peroxisome proliferator-activated receptor *γ* coactivator 1*α* (PGC-1*α*), and inhibit the transcription of CYP7A1 and CYP8B1. In the intestine, FXR induces FGF15/19 to interact with the FGFR4/*β*-Klotho complex on the plasma membrane of liver cells and then initiates extracellular signal-regulated kinase 1/2 (ERK1/2) and Jun-N-terminal kinase (JNK) signaling pathways, which inhibits CYP7A1 expression and BA production. In addition, a recent study showed that the FXR-mediated transcriptional repressor, V-maf avian musculoaponeurotic fibrosarcoma oncogene homolog G (MAFG), can directly inhibit BA synthesis-related genes such as CYP8B1 and regulate BA composition, which may have a significant impact on liver metabolism and related disease [47, 48].

RETRACTED

### 2.5. BAs in the Brain

Cholesterol is a critical component of neurogenesis, and the brain contains more cholesterol than any other organ. Both conjugated and unconjugated BAs can be detected in the brain of humans and rodents [49, 50]. Current studies found that 20 BAs were detected in the rat brain, of which CDCA presented the highest concentration. The BA synthesis pathway in the brain is catalyzed by neuron-specific sterol 24-hydroxylase (CYP46A1) to convert cholesterol into 24(*S*)-hydroxycholesterol [51] (shown in Figure 3). In rat brain, 24(*S*)-hydroxycholesterol can be converted to 3*β*, 7*α*-dihydroxy-5-cholenoic acid or 7*α*-hydroxy-3-oxo-4-cholenoic acid and finally generated CDCA. BAs in the brain mainly come from the synthesis in the brain or transported by brain BA transporters from the peripheral circulation to the brain through the blood-brain barrier (BBB). The unconjugated BAs are lipophilic and therefore, they can cross the BBB mainly by passive diffusion. In contrast, the conjugated BAs have a larger molecular weight and are negatively charged. They require active transport across the BBB via transporters. At present, transporters, such as NTCP, OATP1, BSEP, and MRP2, have been found in choroid plexus and brain capillaries, which can both absorb and excrete BA [52–55].

## 3. BA Activated Receptors

BA homeostasis is regulated by the specific receptors and transporters located in the liver and intestine. There are mainly two kinds of BA–activated receptors [56, 57]: the nuclear receptors and the membrane receptors. The nuclear receptors include FXR, the pregnane X receptor (PXR), and the vitamin D receptor. The membrane receptor contains Takeda G-protein-Coupled receptor 5 (TGR5) and sphingosine-1-phosphate receptor 2 (S1PR2). These receptors play a corresponding regulatory role by binding with BAs which participate in multiple physiological processes such as lipid, glucose, and energy metabolism which expand the important physiological roles of BAs.

### 3.1. Farnesoid X Receptor

FXR, first discovered by Forman et al., in 1995, is a transcription product of NR1H4 [58]. FXR is involved in the biosynthesis of cholesterol, BAs, sterol compounds, porphyrin, ubiquinone, carotenoid, retinoic acid, vitamin D, and steroid hormones. It is considered the master regulator of BA homeostasis. FXR can be activated by BAs in tissues that express BA transporters, such as the terminal ileum, liver, and kidney. CA, CDCA, and its conjugated forms like TCDCA (half of the maximum effective concentration (EC50) =17 *μ*M) are the most potent natural agonists. In the liver and intestine, FXR acts as a BA sensor to negatively inhibit the expression of CYP7A1 and CYP8B1 through the FXR/FGF19/FGFR4 pathway [14] and the hepatic FXR/SHP pathway, respectively. In addition, FXR also regulates BA transporters related to the enterohepatic circulation [59]. In the liver, activated FXR stimulates the excretion of BAs by inducing the expression of carrier proteins BSEP and MDR2/3, which are involved in the streaming of the bile salts and phosphatidylcholine into the biliary duct. In the ileum, activated FXR induces the expression of IBABP, which binds to BAs and facilitates BA transportation in the small intestine. Meanwhile, the OST*α*/OST*β* expression was promoted, and BA was reabsorbed into the portal vein. Moreover, FXR can inhibit BA liver reabsorption by downregulating the expression of liver reabsorption transporter NTCP via SHP dependent mechanism [60]. FXR plays a key role in BA synthesis and enterohepatic circulation. Recent studies have shown that FXR may be a potential therapeutic target for BA metabolism-related diseases such as cholestasis, nonalcoholic fatty liver disease, and type 2 diabetes mellitus [61–63].

RETRACTED

### 3.2. Pregnane X Receptor and vitamin D Receptor

Pregnane X receptor (PXR) is mainly distributed in the small intestine. As a receptor of LCA, it is crucial for the metabolism of toxic LCA in the small intestine. PXR can bind to and be activated by y 5*β*-cholestane-3*α*, 7*α*, 12*α*-triol, and LCA. Activated PXR promotes the 6-hydroxylation of LCA by activating the cytochrome P450-3A (CYP3A) expression and increases the water solubility of LCA, thus reducing its toxicity [64, 65]. Vitamin D receptor (VDR) is expressed in hepatic stellate cells and intestines. LCA was found to be 10 times more sensitive to VDR than PXR. VDR-/- in the intestine can reduce the expression of CYP3A and inhibit the metabolism of LCA [66]. Meanwhile, it can indirectly upregulate the expression of BA transporter, promote the enterohepatic circulation, and transport many toxic BAs to the liver, resulting in liver cholestasis and hepatotoxicity [67].

### 3.3. Takeda G Protein-Coupled Receptor 5

TGR5 is a transmembrane G-protein-coupled receptor (GPCR) for BAs that is widely expressed in the epithelial cells of multiple tissues, including in the intestine, spleen, cholangiocytes, gallbladder, hepatic sinusoidal endothelial cells, and hepatic macrophages [56]. TGR5 can be activated by a variety of BAs, of which LCA, (EC50 = 0.3 *μ*M) is the most potent natural agonist. TGR5 plays an important role in physiology and metabolism. TGR5-related signaling regulates glucose tolerance, inflammation, and energy expenditure and is now considered a potential target for the treatment of metabolic disorders [68, 69]. In addition, recent studies have found that 6-ethyl-23 (S)-methylcholic acid (INT-777), a specific G-protein-coupled BA receptor (TGR5) agonist, has potential neuroprotective effects against LPS-induced cognitive impairment, neuroinflammation, apoptosis, and synaptic dysfunction in mice [70, 71]. Activation of TGR5 may be a new and promising strategy for the treatment of neurological disorders.

RETRACTED

### 3.4. Sphingosine-1-Phosphate Receptor 2

Sphingosine-1-phosphate receptor 2 (SIPR2) is mainly expressed in liver cells like hepatocytes, hepatic stellate cells (HSCs), and hepatic myofibroblast (MFs), and tauro-conjugated BAs are activators of S1PR2 [56, 72, 73]. Recent studies have also found the expression of SIPR2 in neurons and macrophages [74, 75]. Activation of S1PR2 can induce multiple downstream signaling molecules like protein kinase B (Akt), ERK1/2, and c-Jun N-terminal kinase (JNK1/2) and regulates hepatic lipid metabolism or inflammatory reaction, etc. [53, 76, 77].

## 4. BAs and Cognitive Dysfunction-Related Diseases

Cognitive dysfunction usually manifests as impairment of one or more aspects of memory, language, visuospatial, execution, computation, understanding, and judgment. Common cognitive dysfunction-related diseases include MCI, AD, DCD, and VD. Although the exact pathogenesis of each disease state varies, there are some commonalities between them, such as neuroinflammation, deposition of A*β* protein, hyperphosphorylation of Tau protein, loss of neurons, and abnormalities in endoplasmic reticulum stress [78–82]. The “gut-brain axis” has led researchers to recognize the profound impact of gut flora and its metabolites on the nervous system [83, 84]. Metabolomics, genomics, and proteomics studies have found that anomalous changes in BA metabolism and BA receptors of the brain in the patients and animal models of various neurodegenerative diseases. Moreover, experts hypothesized that the alteration of the gut microbiota and subsequent changes in both the serum and brain BA profiles are mechanistically involved in the development of dysfunction-related diseases [85, 86]. Below is recent research highlighting BA signaling and its therapeutic potentials in these cognitive dysfunction-related diseases.

### 4.1. Mild Cognitive Impairment

MCI is an intermediate state between normal aging and dementia. The core symptom of MCI is the decline of cognitive function, which may involve one or more of memory, executive function, language, application, and visual-spatial structure skills, depending on the cause or location of brain damage. It is a neurodegenerative disease commonly seen in the elderly population, which is the preclinical stage of AD. MCI patients are 10 times more likely to develop AD than normal older adults. Due to the lack of effective drugs to prevent or delay the progression of AD, early diagnosis and intervention for MCI patients have become an important means to deal with AD. A targeted metabolomic profiling study revealed that the proportion of serum primary and secondary (both unconjugated and conjugated) BAs was significantly associated with cognitive decline. Compared with the non-MCI group, serum CA levels were decreased, and cytotoxic DCA and GLCA levels were increased. In addition, higher ratios of GDCA: CA and TDCA: CA were observed in MCI patients [87]. What is more, several other studies of serum metabolomics in patients with MCI and AD have found that some certain BAs such as GCA, DCA, GDCA, GCDCA, and LCA were able to distinguish patients with MCI from non-MCI with satisfactory sensitivity and specificity [13, 88, 89]. These findings suggested that the absolute level or relative ratio of certain serum BAs can be used as an early predictor of cognitive decline or the risk of MCI or even AD transformation in patients.

RETRACTED

### 4.2. Alzheimer's Disease

AD is the most common form of dementia, which may lead to personality changes associated with inappropriate emotional and social behavior and cognitive decline. Its main pathological features are senile plaques formed by the deposition of amyloid *β*-protein (A*β*) and nerves formed by hyperphosphorylation of Tau protein fiber entanglement. The causes and mechanisms of AD are complicated. With continuous studies, it is considered that the main pathogenesis of AD includes the degeneration of A*β* [90–92], hyperphosphorylation of Tau protein [93], the imbalance of choline [94], neuroinflammation [95, 96], abnormalities in neurotransmitters, and dysfunction of mitochondrial autophagy [97, 98]. In addition, recent studies have revealed that gut microbiota dysregulation [99, 100] and Ca2+ influx [101, 102] are also closely associated with AD.

The role of BAs in the occurrence and development of AD is an emerging topic. As abnormal alteration in BAs and their receptors have been observed in AD patients, BAs and their receptors have received extensive attention from researchers as biomarkers and potential targets for the diagnosis and treatment of AD. In the latest large-scale clinical study [103], researchers conducted three experiments to investigate whether abnormal cholesterol catabolism, through its conversion into BAs, is associated with the progression of AD and VD. First, they examined serum concentrations of CA, CDCA, and 7*α*-OHC in more than 1,800 participants from two prospective studies and used linear regression and mixed-effects models to examine their association with brain amyloid accumulation white matter lesions and brain atrophy. The results showed that lower serum CA and CDCA concentrations were associated with faster brain atrophy in male patients (FDR *P* = 0.049). In the second study, more than 26,000 patients from the general clinic were studied to explore whether exposure to cholesterol drugs can block the absorption of BAs into the bloodstream, thereby increasing the risk of AD. Results showed that the use of BA blocking drugs significantly increases the risk of dementia in male than female patients. Finally, they examined 29 autopsy samples from AD patients. They found that CA and CDCA were detectable in postmortem brain tissue and were slightly higher in AD patients than in healthy subjects. In addition, there were sex-specific differences in the gene expression of BA receptor neurons in AD. Other metabolomics studies of AD patients or animal models have also shown significant differences in the types and amounts of BAs in AD serum and brain tissue compared with healthy subjects [12, 13, 88, 104–106]. All these founding suggested that abnormal BA metabolism may be one of the causes of cognitive dysfunction in AD, and the change of abnormal BAs' content in serum can be used as one of the biomarkers for the early diagnosis of AD.

RETRACTED

Supplementary of some specific BA like UDCA and TUDCA has been proved to attenuate amyloid precursor protein processing and A*β* deposition, inhibit A*β*-induced synaptic toxicity, reduce neuroinflammation, and improve mitochondrial function in APP/PS1 mice or neurons [107–110]. In an AlCl3-induced AD model, CDCA treatment could ameliorate neurotoxicity and cognitive deterioration via enhanced insulin signaling in rat hippocampus by decreasing the phosphorylation of insulin receptor substrate ser307 (PSER307-IRS1), activating cAMP response element-binding protein (CREB), and enhancing brain-derived neurotrophic factor (BDNF) [111]. The expression of TGR5 in the hippocampus and prefrontal cortex was downregulated in mice with A*β*, lipopolysaccharide (LPS), or streptozocin- (STZ-) induced cognitive dysfunction. INT-777, a selective agonist of TGR5, significantly improved cognitive dysfunction, neuroinflammation, apoptosis, and synaptic damage in these model mice and increased TGR5 expression in the hippocampus and prefrontal cortex [70, 71]. Taken together, data have revealed that BAs and BA signaling are involved in the pathogenesis of AD, and targeting BAs and associated signaling pathways will be promising therapeutic options for the treatment of AD.

### 4.3. Hepatic Encephalopathy

Hepatic encephalopathy (HE) is a serious neurological complication of acute and chronic liver failure. The main clinical manifestations of HE are a disturbance of consciousness, cognitive dysfunction, abnormal behavior, and coma. HE can be caused by a variety of factors, such as oxidative stress, impaired energy metabolism of the brain, impaired blood-brain barrier (BBB) permeability, inflammation, and neurotoxins [112].

RETRACTED

The development of hepatic encephalopathy is a multifactorial process in which altered BA metabolism and signaling due to liver failure are considered as an important risk factor. In a recent large-scale metabolomic study of patients with HE, increased BAs, particularly taurocholic acid and glycolic acid, were detected in the cerebrospinal fluid [113]. Similarly, increased total BA content in brain tissue has been detected in a rodent model of HE [114, 115]. Moreover, the increased total BA content in brain tissue was found before the onset of HE in animal models of liver injury [116], suggesting that BA may play a key role in the pathogenesis of HE. Since only a few certain types of BA can be synthesized in the brain, the high levels of BAs found in the brain tissues of patients with HE may be derived from peripheral circulation and entering the brain through the BBB. Although the mechanism of how BAs enter the brain and are present in cerebrospinal fluid is not fully understood. Studies have found that some BAs may show increased BBB permeability both in vitro and in vivo through Rac1-dependent phosphorylation mechanisms of tight junction protein [117], which may be related to the activation of FXR and TGR5 [118–120]. In addition, another BA activator S1PR2 has been confirmed to regulate BBB permeability by the destabilization of adherens junctions [75, 76, 115]. BAs may regulate BBB permeability by activating S1PR2, but further research is needed. Moreover, BAs can also enter the brain by active transport via apical sodium-dependent BA transporters (ASBT) [121].

Neuroinflammation is another important pathogenesis of HE, in which the activation of microglia acts as a key link [122] (more details are shown in Figure 3). Recent studies have found that proinflammatory chemokine ligand 2 (CCL2) in neurons was increased accompanied by a decrease in the anti-inflammatory chemokine fractalkine in a HE mouse model, resulting in a disruption of the balance between pro- and anti-inflammatory signals acting on microglia, leading to the microglia activation [123, 124]. Interventions targeting BAs and their receptors can attenuate or inhibit microglial activation. For example, administration of BA sequestrant cholestyramine can attenuate microglial activation and reduce BA accumulation in the serum and brain [114]. In addition, S1P2R antagonists can inhibit microglial activation, pro-inflammatory cytokine expression, and subsequent nerve damage associated with HE. However, specific knockdown of FXR in the neuronal cell did not affect microglial activation, suggesting that BA may regulate neuroinflammatory processes by activating S1P2R rather than FXR [115]. The activation of microglia by BA and S1P2R is not directly acted on microglia but through signal transduction communication between neurons and microglia, which is mediated by CCL2. This was confirmed by the specific expression of S1P2R in neurons and treatment of primary microglia with the BA taurocholic acid did not alter the activation state of these cells [115]. In contrast to S1P2R, TGR5 showed a neuroprotective effect which treatment of neurons with TGR5 agonists inhibited microglial activation. Similarly, the TGR5-mediated inhibition of microglia activation is also achieved by inhibiting the CCL2 expression [118], rather than directly acting on microglia.

RETRACTED

### 4.4. Huntington's Disease

Huntington's disease (HD) is an autosomal dominant neurodegenerative disorder. It is caused by amplified mutations of CAG triplet repeats in exon 1 of the Huntingtin (HTT) gene and is often associated with involuntary dance movements, mental and behavioral disorders, and impaired cognitive function [125]. Progressive dementia is an important characteristic of HD. Cognitive dysfunction appears in the early stages of HD. It began with a decline in memory and numeracy in daily life and work. Patients had only mild impairment in remembering new information, but significant deficits in the recall. Cognitive impairment often worsens as the disease progresses. However, unlike AD and other forms of dementia, patients may still retain some cognitive function in the middle and later stages of HD [126]. Impaired cholesterol biosynthesis in rodent HD models and HD patients' fibroblasts and postmortem brains had been reported previously. Levels of cholesterol precursors lanosterol and lathosterol (the whole body cholesterol synthesis index), BA precursor 27-hydroxycholesterol, and brain-specific 24S-hydroxycholesterol (24OHC) were significantly reduced in HD patients' plasma at different disease stages, indicating impaired cholesterol homeostasis in the brain and the whole body [127]. Neuroprotective TUDCA has been shown to reduce 3-nitropropionic acid- (3-NP-) mediated striatum neuronal cell death [128]. In addition, striatal atrophy and apoptosis were significantly reduced in R6/2 transgenic HD mice treated with TUDCA as well as fewer and smaller size ubiquitinated neuronal intranuclear huntingtin inclusions [129].

RETRACTED

### 4.5. Diabetic Cognitive Dysfunction

Diabetic cognitive dysfunction (DCD) is a common neurological complication of diabetes. Patients with diabetes are associated with an increased risk of cognitive impairment, age-related cognitive decline, and dementia [82, 130, 131]. The 2021 American Diabetes Association (ADA) guidelines explicitly address the importance of recognizing cognitive impairment in diabetes and identifying poor glycemic control and recognition [132]. According to the DCD development process or severity, it can be divided into asymptomatic preclinical MCI stage and dementia stage [133]. At present, the mechanism of DCD remains unclear. Studies have shown that insulin resistance may be closely related to the pathogenesis of DCD. In addition, there are other series of hypotheses, including alteration in brain structure and cerebral blood flow, metabolism disorder of neuronal cells, impaired insulin signaling, immune disorders, and mitochondrial dysfunction, and these pathophysiological changes further led to a nerve cell structure and function that is impaired, which affect cognitive function [134–137].

In recent years, it has been found that the abnormal metabolism of BAs may be one of the important pathogenesis of DCD. A previous study conducted by our team on serum metabonomics of DCD patients showed that serum GCA, TCA, and CA levels of DCD patients were significantly changed compared with diabetic patients without cognitive impairment and the healthy people [138]. What is more, similar results have been found in animal models of DCD. The DCD mice exhibited a higher concentration of total BAs in both liver and ileum than unDCD mice. Consequently, DCD mice had increased basolateral BA efflux (Ost*α*, Ost*β*, and MRP4) and decreased BA synthesis (CYP7A1, CYP8B1, and CYP7B1) in the liver as well as activated FXR-FGF15 signaling in the ileum. DCD mice also had increased BA hydroxylation (CYP3A11) and BA sulfation (Sult2a1) in the liver compared to high-fat diet mice. Moreover, these changes were significantly correlated with alterations in gut microbiota [139].

## 5. Conclusions

In summary, most of the previous studies about BA were focused on its physiological role in glucose and lipid metabolism as an endogenous metabolite and signal molecule. In recent years, the role of BAs and targeting bile acid-mediated signaling in the treatment of cognitive disability-related diseases has been gradually identified. Most of the studies have focused on the neuroprotective effects of certain BAs like UDCA and TUDCA and have been well demonstrated in cellular and animal models and human clinical trials. However, due to the BAs being a relatively large group of structurally related molecules, little is known about the potential efficacy of other types of BAs in cognitive dysfunction-related diseases. Although current studies have found that BAs and their receptors, such as TGR5, FXR, and SIPR2, are abnormally altered in cognitive dysfunction-related diseases, two issues remain to be addressed. One is the precise information of changes in the BA profiles in the blood or brain and its correlation with the degree of cognitive dysfunction. This will provide important guidance for the utilization of BAs as a predictive or diagnostic indicator of these diseases. The other is to determine the precise molecular mechanisms of neurotoxicity or neuroprotective effects by BAs their receptors in cognitive dysfunction-related diseases, which will provide a theoretical basis for the novel discoveries and strategies for the prevention and treatment of cognitive dysfunction related disease.

RETRACTED

## Figures and Tables

**Figure 1:** Bile acid synthesis and metabolism. BAs are synthesized in the perivenous hepatocytes through a series of enzymatic reactions. There are the classical and alternative pathways for bile acid synthesis: The “classic pathway” is formed by a series of catalytic reactions via CYP7A1, HSD3B7, CYP8B1, and CYP27A1. Two hydrophobic primary bile acids, CA and CDCA, were synthesized. CYP7A1 located in the endoplasmic reticulum of liver cells is the main rate-limiting enzyme in this pathway. The alternative pathway occurs in a variety of tissues and macrophages, which is initiated by CYP27A1 in mitochondria and CYP7B1 in the endoplasmic reticulum to synthesis CDCA. In the rodent liver, primary bile acids *α*- and *β*-MCA are generated by 7*β*-hydroxylation from CDCA and UDCA via CYP2C70. Primary BAs are then combined with glycine or taurine to form conjugated BAs. The conjugated BAs were transported from liver cells to the gallbladder by BESP and MRP2. After eating, the gallbladder contracts and secretes BAs into the intestine. Primary BAs are metabolized by intestinal bacteria to produce secondary BAs, mainly including DCA, LCA, and HDCA.

**Figure 2:** The enterohepatic circulation and negative feedback regulation mechanism of BAs. At the terminal ileum, about 95% of unconjugated BAs are actively ingested through the ASBT at the tip of the brush edge of the small intestine and then enter the small intestinal epithelial cells. After binding with the IBABP, BAs are secreted into the portal vein by the OST*α*/OST*β*. Then, the BAs are reabsorbed by liver cells via NTCP and OATPs. In addition, a small amount of BAs in the liver can also enter the peripheral circulation through MRP3, MRP4, and the OST*α*/OST*β* complex. The biosynthesis is regulated by a negative feedback mechanism through three ways: ① in the liver, excess BA activates FXR, which induces the expression of the target gene SHP. SHP inhibits the gene expression of CYP7A1 and CYP8B1 and reduces BAs production by binding with LRH-1. ② In intestine, FXR induces FGF15/19 to interact with the FGFR4/*β*-Klotho complex on the plasma membrane of liver cells and then initiates ERK1/2-JNK signaling pathways, which inhibits CYP7A1 expression and BA production. ③ FXR-mediated transcriptional repressor, VMAFG, can directly inhibit BA synthesis-related gene CYP8B1 and regulate BA synthesis.

RETRACTED

**Figure 3:** BA metabolism in the brain and its association with cognitive dysfunction-related diseases. In the brain, cholesterol is oxidized to 24-OH via CYP46A1. The 24-OH can easily exit the brain through the ABCA1. This is the main way of cholesterol clearance in the brain. ① In AD, the BBB is broken due to the hydrophobic environment created by an increase in blood lipids (hyperlipidemia and hypercholesterolemia), which allows toxins produced by the gut flora to penetrate the brain. Secondary BAs damage neurons that produce CYP46A1, simultaneously activating FXR and reducing the expression of CYP46A1. As a result, the cholesterol clearance pathway in the brain is disrupted, and the high-cholesterol environment in the brain positively regulates *β*- and *γ*-secretase expression, increasing the amyloid protein production pathway, leading to the deposition of A*β* in the brain. ② In addition, neuroinflammation caused by activation of microglia in HE is thought to be closely associated with the development of cognitive dysfunction. Specific conjugated BAs in the brain induce microglial activation and secrete proinflammatory factors by activating S1P2R. This process is not directly acted on microglia but through signal transduction communication between neurons and microglia, which is mediated by CCL2.

**Table 1:** The main bacterial genera of the gut microbiota involved in BA metabolism.

Function	Bacterial genera	References
BSH deconjugation	*Bacteroides*, *Clostridium*, *Lactobacillus*, *Bifidobacterium*, and *Listeria*	[29, 30]
Oxidation and epimerization of hydroxyl groups at C3, C7, and C12	*Bacteroides*, *Eubacterium*, *Clostridium*, *Escherichia*, *Eggerthella*, *Peptostreptococcus*, and *Ruminococcus*	[31–33]
7*α*-Dehydroxylation	*Clostridium* and *Eubacterium*	[34–36]
Esterification	*Bacteroides*, *Eubacterium*, and *Lactobacillus*	[37, 38]
Desulfation	*Clostridium*, *Fusobacterium*, *Peptococcus*, and *Pseudomonas*	[10, 14, 39]
